# The Tet2–Upf1 complex modulates mRNA stability under stress conditions

**DOI:** 10.3389/fgene.2023.1158954

**Published:** 2023-04-06

**Authors:** Meiling Xia, Rui Yan, Wenjuan Wang, Anqi Kong, Meng Zhang, Zhigang Miao, Wei Ge, Bo Wan, Xingshun Xu

**Affiliations:** ^1^ Departments of Neurology, The Second Affiliated Hospital of Soochow University, Suzhou, China; ^2^ Institute of Neuroscience, Soochow University, Suzhou, China; ^3^ Department of Neurology, The Affiliated Hospital of Xuzhou Medical University, Xuzhou, China

**Keywords:** Tet2, Upf1, RNA, 5hmC, mRNA stability

## Abstract

**Introduction:** Environmental stress promotes epigenetic alterations that impact gene expression and subsequently participate in the pathological processes of the disorder. Among epigenetic regulations, ten–eleven Translocation (Tet) enzymes oxidize 5-methylcytosine (5mC) to 5-hydroxymethylcytosine (5hmC) in DNA and RNA and function as critical players in the pathogenesis of diseases. Our previous results showed that chronic stress increases the expression of cytoplasmic Tet2 in the hippocampus of mice exposed to chronic mild stress (CMS). Whether the cytoplasmic Tet2 alters RNA 5hmC modification in chronic stress-related processes remains largely unknown.

**Methods:** To explore the role of cytoplasmic Tet2 under CMS conditions, we established CMS mice model and detected the expression of RNA 5hmC by dot blot. We verified the interaction of Tet2 and its interacting protein by co-immunoprecipitation combined with mass spectrometry and screened downstream target genes by cluster analysis of Tet2 and upstream frameshift 1 (Upf1) interacting RNA. The expression of protein was detected by Western blot and the expression of the screened target genes was detected by qRT-PCR.

**Results:** In this study, we found that increased cytoplasmic Tet2 expression under CMS conditions leads to increase in total RNA 5hmC modification. Tet2 interacted with the key non-sense-mediated mRNA decay (NMD) factor Upf1, regulated the stability of stress-related genes such as Unc5b mRNA, and might thereby affect neurodevelopment.

**Discussion:** In summary, this study revealed that Tet2-mediated RNA 5hmC modification is involved in stress-related mRNA stability regulation and may serve as a potential therapeutic target for chronic stress-related diseases such as depression.

## Introduction

Epidemiological studies have revealed that chronic stress caused by environmental factors has a significant impact on diseases (Jirtle and Skinner, 2007; Burrage et al., 2018; Wen-Yue and Xiao-Dong, 2021). Adverse experiences, such as emotional abuse (LeMoult et al., 2020), isolation (Slavich and Sacher, 2019), smoking (Fluharty et al., 2017), alcoholism (Schuckit, 2009), and obesity (Milaneschi et al., 2019), are highly sensitive to environmental stress, especially during early life, a critical period of brain developmental plasticity. These environmental stress factors influence an individual’s genome through inducing changes in epigenetic modifications and are high-risk factors for psychiatric disorders such as depression (Green et al., 2010; Barbu et al., 2021).

Chronic environmental stress induced several types of epigenetic modifications to regulate gene expression in the pathological process of depression (Dalton et al., 2014; Mayer et al., 2021). For instance, people with major depressive disorder (MDD) showed a decreased global DNA 5hmC in peripheral leukocytes (Tseng et al., 2014; Reszka et al., 2021). Some antidepressants also showed the effect of increasing the level of DNA 5hmC (Wei et al., 2014; Wang et al., 2019). Therefore, as the dioxygenase of DNA or RNA 5-methylcytosine (Ito et al., 2010; Fu et al., 2014; Lan et al., 2020; Ma et al., 2022), the Tet family may be one of the genetic modifiers responsible for MDD. The Tet family includes three members: Tet1, Tet2, and Tet3 (Rasmussen and Helin, 2016). Our previous study found that the expression of Tet2 increased in the hippocampus of mice after chronic stress and Tet2 mainly accumulated in the cytoplasm (Zhang et al., 2021). However, the role of Tet2 accumulation in the cytoplasm under stress conditions remains unclear.

Recent studies have shown that methylation and demethylation modifications were also found in RNA cytosine, namely, RNA 5mC and RNA 5hmC (Motorin et al., 2010). These modifications are involved in RNA processing (Yang et al., 2017), mRNA stability (Chen et al., 2019; Yang et al., 2019), neural system development (Flores et al., 2017), and tumorigenesis (Liang et al., 2020). Tet enzymes, such as the dioxygenase of DNA 5mC (Tsiouplis et al., 2020), have also been found to serve as the hydroxymethylase of RNA 5 mC (Fu et al., 2014; Guallar et al., 2018). The ATP-dependent RNA helicase upstream frameshift 1 (Upf1) has potential interactions with Tet2 protein according to the mass spectrometry result of Tet2 protein. Upf1 impacts mRNA stability (Staszewski et al., 2023) and is the most enriched RNA-binding protein of the 5mC site in mRNA (Amort et al., 2017). Whether Upf1 participates in the Tet2-mediated hydroxymethylation of RNA 5mC is still unknown.

In this study, we found that the expression of RNA 5hmC modification increased under CMS conditions accompanied with increased cytoplasmic Tet2. The ATP-dependent RNA helicase Upf1 was identified as a Tet2-interacting protein to modify RNA 5hmC and regulate RNA stability such as Unc5b mRNA, which is involved in axonal guidance and stress responses. Our findings, therefore, provide novel mechanistic insights into the role of epigenetic modification induced by Tet2 in chronic stress, suggesting the pathological importance of cytoplasmic Tet2 and RNA 5hmC modification in psychiatric disorders.

## Materials and methods

### Reagents, antibodies, cell lines, and oligos

The lists of the reagents, antibodies, cell lines, and oligos used in this study are given in Supplementary Table S1.

### Animals and establishment of chronic mild mice model

All procedures and protocols in this study were approved by the Institutional Animal Care and Use Committee of Soochow University. C57BL/6 mice (25.0 ± 3.0 g, 8–12 weeks old) were purchased from the Shanghai Research Center for Model Organisms. The mice were randomly divided into two groups: the control group and the model group and exposed to various, randomly scheduled, low-intensity social and environmental stressors two–three times a day for 5 weeks. The stressors included the following: (Jirtle and Skinner, 2007) water deprivation for 24 h, (Wen-Yue and Xiao-Dong, 2021) food deprivation for 24 h, (Burrage et al., 2018) wet cage for 24 h, (LeMoult et al., 2020) empty cage for 24 h, (Slavich and Sacher, 2019) cage tilt for 24 h (45°), (Fluharty et al., 2017) restraint stress for 2 h, (Schuckit, 2009) forced swimming at 4°C for 6 min, (Milaneschi et al., 2019) cage exchange for 6 min, (Green et al., 2010) shaking the cage for 6 min, (Barbu et al., 2021) and giving noise for 6 min. The control mice were housed under normal conditions (four to five per cage) and only switched to individual housing during testing for the depressive-like behavior phase.

### Tail suspension test (TST)

Depression in mice was assessed using the TST (Sidransky et al., 2009). First, the mice were suspended 55 cm above the floor with a medical tape placed about 2 cm from the tip of their tails. The mice were made to turn to the camera to prevent them from being affected by the camera. The immobility time of the mice was recorded using a video camera for 6 min. The criterion for mouse immobility was immobility for at least 2 s.

### Forced swimming test (FST)

The FST was used to assess mice for depressive behavior. The FST apparatus consisted of a transparent glass cylinder (18 cm diameter and 40 cm height) filled with water up to 15 cm at about 25°C. The cylinder was wrapped in tin foil paper to prevent interference while the mice swam. Pre-testing is required before a formal experiment. Mice were placed in a cylinder and allowed to swim and then removed from the water and returned to the cage after been dried in a heated environment for several minutes. In the formal test, the camera was placed directly above the cylinder, and the immobility time of the mice was measured during a 6-min swim after being placed in the water. At the end of each test, the warm water should be refilled so as not to affect the subsequent measurement tests. The criterion for immobility in mice is to stay afloat without struggling.

### Sucrose preference test (SPT)

In this test, mice with anhedonia were evaluated with reference to the method of Liu et al., (2018) mentioned in published articles. Before the test, the mice were acclimated to the cage with two randomly placed tubes containing 1% (w/v) sucrose solution and water for 3 days. During the adaptation period, new tubes will be replaced daily, and the tube is placed at random positions each day. In the SPT, mice could prefer to drink 2% (w/v) sucrose solution or water freely, and the volume of sucrose solution or water was recorded at the second hour and the 24th hour, respectively. The sucrose preference is calculated using the following equation: ratio of sucrose preference = consumption of sucrose/[consumption of water + consumption of sucrose] × 100%.

### Cell culture and transfection

Neuro 2A (N2a) cells and HEK293T cells were cultured in Dulbecco’s modified Eagle’s medium (DMEM) supplemented with 10% fetal bovine serum (FBS) and were placed in a humidified incubator at 37°C with 5% CO_2_. For transfection, HEK293T cells were transfected at 70% confluency using polyethylenimine (PEI), and N2a cells were transfected at 70% confluency using PL transfection reagent according to the manufacturer’s instructions.

### Immunoprecipitation (IP), protein extraction, and Western blot

For endogenous IP, three 90-mm dishes containing N2a cells at 70% confluency were lysed in 1 mL RIPA buffer [50 mM Tris (pH 8.0), 0.1% SDS, 150 mM NaCl, 1 mM EDTA (pH 8.0), 1 mM EGTA (pH 8.0), 0.5% deoxycholate, and 1% Triton X-100] containing 100 × cocktail and 200 × DTT at 4°C under rotary agitation for 30 min. About 5% input was taken after centrifuging at 13,200 rpm for 30 min at 4°C. Total protein was divided into two groups, and each group contained not less than 2 mg. The protein supernatant was added after agarose beads were activated and was pre-cleared by rotating for 2 h at 4°C. The supernatant was transferred to another tube, and the same amount of Tet2 and IgG antibody was added into the two tubes and then rotated at 4°C overnight. The supernatant was transferred to the agarose beads and rotated at 1,000 rpm at 4°C overnight. The supernatants were removed after centrifuging at 1,000 rpm at 4°C for 3 min, 50 μL 2 × loading buffer was added to the precipitate, and the samples were boiled at 95°C for 10 min.

For exogenous IP, HEK293T cells were transiently transfected with target plasmids using PEI. Three 90-mm dishes of HEK293T cells were used as one group. HA-Upf1 (30 μg) + Vector (30 μg) and HA-Upf1 (30 μg) + Flag-Tet2 (30 μg) plasmids were transfected for 48 h. Cell pellets were lysed using lysis buffer [150 mM NaCl, 25 mM tris-HCl (pH 7.4), 10% glycerol, 0.5% Triton X-100, 2 mM MgCl_2_] containing 100 × cocktail and 200 × DTT at 4°C for 30 min; centrifuged at 4°C for 30 min at 13,200 rpm; and 60 μL of the supernatant was collected as the input sample. The remaining supernatant was put into Flag beads and rotated at 4°C overnight. The supernatant was removed by a magnetic shelf, and the beads were cleaned twice with lysis buffer. About 50 μL 1 × loading buffer was added to the precipitate, and the samples were boiled at 95°C for 10 min.

For total protein extraction, cell pellets were lysed using RIPA buffer containing 50 mM Tris (pH 8.0), 0.1% SDS, 150 mM NaCl, 1 mM EDTA (pH 8.0), 1 mM EGTA (pH 8.0), 0.5% deoxycholate, and 1% Triton X-100 on ice for 30 min and then centrifuged at 4°C at 12,000 rpm for 15 min. The supernatant was collected and boiled for 10 min at 95°C after adding 1/4 volume of 5 × loading buffer. About 30-μg protein aliquot of each sample was separated using standard SDS-PAGE and transferred onto a PVDF membrane. After transferring the protein, the PVDF membrane was blocked with 10% nonfat milk for 1 h at room temperature (RT) and incubated overnight at 4°C with target primary antibody. Immunoreactive bands were detected by ECL chemiluminescence reagent after incubating with secondary antibody for 1 h. The antibody and reagents used in this experiment are given in the Supplementary Material.

### Immunofluorescence

The samples were fixed overnight at 4°C in 4% PFA in PBS for 30 min, treated with 0.3% Triton X-100 in PBS (PBST) for 10 min, and then blocked with 5% BSA in 0.3% PBST for 1 h at RT. Subsequently, the samples were incubated with sample-specific primary antibodies overnight at 4°C, followed by three washes with PBS, and incubated with florescent-labeled secondary antibody containing DAPI for 1 h at RT. The samples were imaged using a fluorescence microscope (Axio Scope A1, Zeiss) after patching on the microslide.

### Construction and transformation of the expression plasmids

RNA was extracted from the hippocampus of wild-type C57BL/6 mice and reverse-transcribed onto cDNA. Target fragments were amplified from this cDNA as templates. The gel extraction products of target fragments were linked with linearized pCMV-HA or pCMV-flag plasmids by homologous recombination. DH5α *E.coli* was used to transform the connection products obtained in the aforementioned experiments. After transformation, monoclonal colony was selected for plasmid amplification. The plasmids were extracted and verified by sequencing.

### Overlapping genes and functional enrichment analysis

The overlapping genes list was obtained from the jvenn database (http://jvenn.toulouse.inra.fr/app/example.html). Metascape (http://metascape.org/gp/index.html#/main/step1) is a gene-list analysis tool for gene functional enrichment analysis (Zhou et al., 2019). The identified overlapping genes were inputted into the Metascape database for Gene Ontology (GO), Kyoto Encyclopedia of Genes and Genomes (KEGG) pathways, and disease enrichment analysis.

### RNA isolation and quantitative RT–PCR

Total RNA was extracted using RNA TRIzol and was reverse-transcribed using the Reverse Transcription Kit as per the manufacturer’s protocol. Quantitative real-time PCR was performed using 2 × SYBR Green PCR Master Mix with a 7500 real-time PCR system (Applied Biosystems, Foster City, CA, United States). GAPDH was used as an endogenous control for real-time PCR amplification. For data analysis, fold change was calculated using the ΔΔCt method according to the threshold cycle (Ct) value obtained from RT-PCR. The sequences of the primers used in this study are given in Supplementary Material.

### RNA isolation and dot blot

Total RNA was extracted using RNA TRIzol and was reverse-transcribed using the Reverse Transcription Kit as per the manufacturer’s protocol. During RNA extraction, DNase I, RNase-free pipettor tips, RNase-free centrifugal tubes, and other RNase-free plastic products were used, and RNA was dissolved in RNase-free water treated by DEPC. After the extraction, the RNA purity was tested using a NanoDrop 2000 spectrophotometer. For dot blot, a 20-μL system containing 2,000 ng RNA, 10 μL 2M NaOH (denature solution), and double distilled water was prepared. Then, the mix was allowed to stand at 4°C for 20 min. We spotted 2 µL of samples onto the nitrocellulose (NC) membrane and allowed the membrane to dry at RT. RNA was fixed to the membrane by incubating at 80°C for 30 min. Then, the NC membrane was blocked with 10% nonfat milk for 1 h at RT and incubated with 5hmC antibody overnight at 4°C. The immunoreactive signal was detected by ECL chemiluminescence reagent after 2-h incubation with secondary antibody at RT. Also, the dot signal was quantified by using ImageJ software.

### Statistical analysis

All statistical analyses were performed using Prism 7.0 (GraphPad Software) and are expressed as means ± SEM. The differences with different treatments were determined by *t*-test or one-way ANOVA, followed by the Tukey’s *post hoc* test, and were considered statistically significant at *p* < 0.05.

## Results

### RNA 5hmC modification and Tet2 expression increased in the hippocampus of CMS mice

Our previous results showed high levels of RNA 5hmC modification in the brainstem, hippocampus, and cerebellum of mice, and RNA 5hmC modification was downregulated in the MPTP-induced mouse model (Miao et al., 2016), but the changes of RNA 5hmC in depressed mice are still unclear. Therefore, by establishing a CMS mouse model (Figure 1), we detected the RNA 5hmC level in the hippocampus and prefrontal cortex, which are most sensitive to the neurotoxic effects of stress (McEwen et al., 2016). Dot blot results showed that the level of RNA 5hmC was increased in the hippocampus (*p* < 0.01, Figures 2A, B) and prefrontal cortex (*p* < 0.05, Figures 2C, D) of CMS mice compared with the control group. Because RNA 5hmC is relatively less distributed in the cortex (Miao et al., 2016), the hippocampal region was selected for further research.

**FIGURE 1:** Establishment and identification of CMS model mice. **(A)** Experimental paradigm of the CMS model. **(B–E)** Behavioral tests were performed after the experimental procedure. **(B)** TST, *n* = 29, 23, ****p < 0.0001. **(C)** FST, *n* = 40, 33, ****p < 0.0001. **(D)** SPT at the second h, *n* = 38, 37, ***p < 0.001. **(E)** SPT at the 24th h, *n* = 31, 33, **p < 0.01. All data are presented as the mean ± S.E.M. Unpaired two-tailed Student’s t-test was used.

**FIGURE 2:** RNA 5hmC modification and Tet2 expression increased in the hippocampus of CMS mice. **(A,B)** Representative dot blot **(A)** and quantitative analysis **(B)** of RNA 5hmC abundance in the hippocampus (HIP) brain regions of control and CMS mice. *n* = 4, **p < 0.01. **(C,D)** Representative dot blot **(C)** and quantitative analysis **(D)** of RNA 5hmC abundance in the brain regions of the prefrontal cortex (PFC) of control and CMS mice. *n* = 4, *p < 0.05. **(E–G)** Quantitative RT-PCR of Tet1 **(E)**, Tet2 **(F)**, and Tet3 **(G)** mRNA levels in the hippocampus of control and CMS mice. *n* = 3, *p < 0.05, **p < 0.01. **(H, I)** Representative Western blot **(H)** and quantitative analysis **(I)** of Tet1 protein levels in the mouse hippocampus. *n* = 3, *p < 0.05. **(J, K)** Representative Western blot **(J)** and quantitative analysis **(K)** of Tet2 protein levels in the mouse hippocampus. *n* = 3, **p < 0.01. **(L,M)** Representative Western blot **(L)** and quantitative analysis **(M)** of Tet3 protein levels in the mouse hippocampus. *n* = 3, **p < 0.01. Quantified data are normalized to the control group, whose value is equal to 1. All data are presented as the mean ± S.E.M. Unpaired two-tailed Student’s t-test was used.

Studies have shown that RNA 5hmC is derived from RNA 5mC and is mainly catalyzed by Tet proteins (Fu et al., 2014). Thus, we detected the expression of Tet proteins including Tet1, Tet2, and Tet3 in the hippocampus of CMS mice. Compared with the control group, the mRNA level (*p* < 0.01, Figure 2F) and protein level (*p* < 0.01, Figures 2J, K) of Tet2 were increased in the hippocampus of CMS mice, while the level of Tet1/Tet3 mRNA (*p* < 0.05, Figures 2E, G), Tet1 protein (*p* < 0.05, Figures 2H, I), and Tet3 protein (*p* < 0.01, Figures 2L, M) significantly decreased. Therefore, this indicated that the increase in RNA 5hmC modification in the hippocampus of CMS mice results from the increase in Tet2, rather than Tet1 and Tet3.

### Tet2 regulated RNA 5hmC levels

To further validate the role of Tet2 in the oxidation of RNA 5mC to 5hmC, we examined RNA 5hmC levels in N2a cells by either Tet2 knockdown or overexpression. Tet2 knockdown markedly decreased Tet2 mRNA and protein expression in N2a cells (*p* < 0.0001, 0.01, Figures 3A–C). At the same time, RNA 5hmC level was significantly reduced in Tet2 knockdown N2a cells (*p* < 0.01, Figures 3D, E). Due to high molecular weight of full-length Tet2, and previous studies having confirmed that the catalytic domain of Tet2 (Tet2 CD) also has the 5mC hydroxymethylation modification function as the full-length Tet2 (Fu et al., 2014), we overexpressed Tet2 CD in N2a cells (*p* < 0.0001, Figures 3F, G). The RNA 5hmC level significantly increased after Tet2 CD overexpression (*p* < 0.05, Figures 3H, I).

**FIGURE 3:** Tet2 regulated RNA 5hmC levels. **(A)** Quantitative RT-PCR of Tet2 mRNA levels in Tet2 knockdown N2a cells. *n* = 5, ****p < 0.0001. **(B,C)** Representative Western blot **(B)** and quantitative analysis **(C)** in Tet2 knockdown N2a cells. *n* = 3, **p < 0.01. **(D,E)** Dot blot quantification of RNA 5hmC abundance before and after Tet2 knockdown. *n* = 4, **p < 0.01. **(F)** Representative images of immunoblots of the transfection efficiency of Tet2 CD in the N2a cells. **(G)** Quantitative analyses of Tet2 mRNA levels before and after overexpression of Tet2 CD. *n* = 3, ****p < 0.0001. **(H,I)** Dot blot quantification of RNA 5hmC abundance before and after Tet2 CD overexpression. *n* = 3, *p < 0.05. Quantified data are normalized to the control group, whose value is equal to 1. All data are presented as the mean ± S.E.M. Unpaired two-tailed Student’s t-test was used.

### The expression of Upf1, a Tet2-interacting protein, increased in the hippocampus of depressed mice

To further investigate the function of Tet2-mediated RNA 5hmC modification, we analyzed the mass spectrometry data of the potential interacting proteins of Tet2 (Guallar et al., 2018) and found that a large portion of the proteins interacting with Tet2 were involved in the mRNA processing pathway (Figure 4A). Among the Tet2-interacting protein candidates, Upf1 was found to potentially interact with Tet2. A previous study showed the Upf1 protein has binding sites that significantly overlap with 5mC sites in mouse embryonic stem cells and brain (Amort et al., 2017). This suggests that 5mC may contribute to the binding and functionality of Upf1. To explore the role of Upf1 in Tet2-mediated RNA hydroxymethylation modification, we co-transfected Flag-Tet2 plasmids with HA-Upf1 plasmids in HEK293T cells and found that HA-Upf1 could be precipitated by Flag-Tet2 (Figure 4B). The interaction was also confirmed with endogenous Tet2 and Upf1 in N2a cells (Figure 4C). In addition, we also observed the colocalization of Tet2 and Upf1 in the cytoplasm of HEK293T cells with Flag-Tet2 and HA-Upf1 overexpression (Figure 4D). Subsequently, we detected the expression of Upf1 in the hippocampus of CMS mice. Our results showed that the expression of Upf1 significantly increased in the hippocampus of CMS mice (*p* < 0.05, 0.001, Figures 4E–G).

**FIGURE 4:** Tet2-interacting protein Upf1 increased in the hippocampus of stressed mice. **(A)** Pathway map of Tet2-interacting proteins constructed by GO gene function analysis. **(B)** Exogenous Co-IP experiment was performed using HEK293T cells. Flag-Tet2 and HA-Upf1 were transfected into HEK293T cells as indicated, and the cell lysates were subsequently immunoprecipitated using anti-Flag. The immunoprecipitates were examined by Western blotting with anti-HA antibody. Input represented 10% of cell lysates used in the Co-IP experiment. **(C)** Endogenous Co-IP experiment was performed using N2a cells. Cell lysates from cells were incubated with anti-Tet2 antibody. For Western blotting of immunoprecipitates, anti-Upf1 antibody was used. **(D)** HEK293T cells were transfected with Flag-Tet2 plasmids and HA-Upf1 plasmids and stained for Flag (red), HA (green), and DAPI (blue). Representative immunofluorescence images revealed the colocalization of Flag-Tet2 and HA-Upf1 in the cytoplasm of HEK293T cells. Scale bar, 25 μm. **(E)** RT-PCR detection of Upf1 mRNA levels in the hippocampus of control and CMS mice. *n* = 3, *p < 0.05. **(F,G)** Western blot detection of Upf1 protein levels in the hippocampus of control and CMS mice. *n* = 3, ***p < 0.001. Quantified data are normalized to the control group, whose value is equal to 1. All data are presented as the mean ± S.E.M. Unpaired two-tailed Student’s t-test was used.

### Downstream genes of the Tet2–Upf1 complex reduced in the hippocampus of stressed mice

In order to investigate the influence of Tet2 and Upf1 on RNA 5hmC modification, we screened candidate downstream target genes of the interaction of Tet2 and Upf1 from the data of Tet2 RNA co-immunoprecipitation (Tet2-RIP) (Lan et al., 2020) and Upf1 RNA co-immunoprecipitation (Upf1-CLIP) (Hurt et al., 2013). GO analysis and cluster analysis of the overlapped genes (Supplementary Table S2) revealed the existence of stress-related pathways such as axonal guidance and neural development (Figure 5A). The potential target genes Ntn1, Unc5b, Ptpn11, and Src are included in this pathway (Figure 5B) and participate in the process of psychiatric disorders such as depression (Zeng et al., 2017; Perrino et al., 2018; Meng et al., 2022). The changes of these target genes under CMS were detected by RT-PCR, and the results showed that the expression of these target genes at the mRNA level was reduced after stress compared with the control group (*p* < 0.05, 0.01, Figures 5C–F). Therefore, we selected Ntn1, Unc5b, Ptpn11, and Src as the candidate genes in this study to explore the effect of the Tet2–Upf1 complex to mRNA stability due to the RNA helicase property of Upf1.

**FIGURE 5:** Downstream genes of the Tet2–Upf1 complex reduced in the hippocampus of stressed mice. **(A)** Screening of intersection target genes using Tet2-RIP and Upf1-CLIP data. **(B)** Screening of stress-related intersection target genes. **(C–F)** RT-PCR detection of the mRNA levels of target genes Ntn1 (*p < 0.05) **(C)**, Unc5b (**p < 0.01) **(D)**, Ptpn11 (*p < 0.05) **(E)**, and Src(*p < 0.05) **(F)** in the hippocampus of control mice and CMS mice. *n* = 5. Quantified data are normalized to the control group, whose value is equal to 1. All data are presented as the mean ± S.E.M. Unpaired two-tailed Student’s t-test was used.

### The target gene Unc5b was significantly altered after Tet2 or Upf1 knockdown

To investigate the mechanism by which the Tet2–Upf1 complex affects downstream target genes, we knocked down Tet2 and Upf1 in N2a cells, respectively (*p* < 0.05, 0.001, Figures 6A–D), and analyzed the expression of target genes Ntn1, Unc5b, Ptpn11, and Src. The results showed that Unc5b had the most significant change in mRNA level after knockdown of Tet2 (*p* < 0.01, Figures 6E–H) and Upf1 (*p* < 0.05, 0.01, Figures 6I–L). Unc5b is involved in many biological processes, including neural development (Boyé et al., 2022), angiogenesis (Potente et al., 2011), tumor processes (Kong et al., 2016), and the occurrence of post-stress depression (Zeng et al., 2017), so we next examined Unc5b RNA 5hmC modification as a representative target gene of the Tet2–Upf1 complex.

**FIGURE 6:** Unc5b reduced after knockdown of Tet2 or Upf1. **(A)** RT-PCR detection of the mRNA level of knockdown Upf1 in the constructed shUpf1-1 plasmid. *n* = 3, *p < 0.05. **(B)** RT-PCR detection of the mRNA level of knockdown Upf1 in the constructed shUpf1-2 plasmid. *n* = 4, ***p < 0.001. **(C,D)** Western blot detection of the protein level of knockdown Upf1 in the constructed shUpf1-2 plasmid. *n* = 3, ***p < 0.001, ****p < 0.0001. **(E–H)** RT-PCR detection of mRNA levels of Ntn1 **(E)**, Unc5b **(F)**, Ptpn11 **(G)**, and Src **(H)** before and after knockdown of Tet2. *n* = 4–6. ns: no significant, **p < 0.01. **(I–L)** RT-PCR detection of mRNA levels of Ntn1 **(I)**, Unc5b **(J)**, Ptpn11 **(K)**, and Src **(L)** before and after knockdown of Upf1. *n* = 3–6. *p < 0.05, **p < 0.01. Quantified data are normalized to the control group, whose value is equal to 1. All data are presented as the mean ± S.E.M. Unpaired two-tailed Student’s t-test was used.

### Tet2–Upf1 complex affects the stability of Unc5b mRNA

Previous studies have demonstrated that RNA 5hmC modification regulates mRNA stability at the post-transcriptional level (Lan et al., 2020). In order to investigate whether Tet2 regulates the stability of Unc5b mRNA through RNA 5hmC modification, we treated the Tet2 knockdown N2a cells with actinomycin D (ActD) to inhibit transcription and examined the Unc5b mRNA stability. The results showed that Tet2 knockdown increased the stability of Unc5b mRNA (*p* < 0.05, Figure 7A). At the same time, we examined the Unc5b mRNA level after overexpression of Tet2 CD, and the results showed that the expression level of Unc5b mRNA decreased after overexpression of Tet2 CD (*p* < 0.01, Figure 7B), and the stability of Unc5b mRNA decreased after Tet2 CD overexpression (*p* < 0.05, Figure 7C). A previous study showed that Upf1 is a major protein involved in regulating mRNA stability [38]. To verify whether Upf1 is also involved in the regulation of Unc5b mRNA stability, we knocked down Upf1 in N2a cells. Upf1 knockdown increased the stability of Unc5b mRNA (*p* < 0.05, Figure 7D). Similarly, the mRNA level of Unc5b decreased after overexpression of Upf1 (*p* < 0.05, Figures 7E, F) and the stability of Unc5b mRNA was decreased after overexpression of Upf1 (*p* < 0.05, Figure 7G). To further verify that Tet2 and Upf1 participate in the regulation of Unc5b mRNA stability through a complex, we co-transfected HA-Upf1 plasmids with siTet2 in N2a cells and detected the Unc5b mRNA level. Our results showed that Upf1 overexpression decreased the Unc5b mRNA expression and stability, while Tet2 knockdown partially rescued the reduction of Unc5b mRNA expression and stability (*p* < 0.01, Figures 7H, I). Taken together, our results suggested that Tet2 and Upf1 have a synergistic effect on Unc5b mRNA stability.

**FIGURE 7:** Tet2–Upf1 complex regulated Unc5b mRNA stability. **(A)** Stability of Unc5b mRNA before and after knockdown of Tet2 was detected by RT-PCR. *n* = 6, *p < 0.05. **(B)** mRNA levels of Unc5b before and after overexpression of Tet2 CD were detected by RT-PCR. *n* = 4, **p < 0.01. **(C)** Stability of Unc5b mRNA before and after overexpression of Tet2 CD was detected by RT-PCR. *n* = 6, *p < 0.05. **(D)** RT-PCR to detect the stability of Unc5b mRNA before and after knockdown of Upf1. *n* = 3, *p < 0.05. **(E)** Western blot to detect the transfection efficiency of HA-Upf1 in N2a cells. **(F)** RT-PCR detection of Unc5b mRNA levels before and after Upf1 overexpression. *n* = 4, *p < 0.05. **(G)** RT-PCR detection of Unc5b mRNA stability before and after Upf1 overexpression. *n* = 6, *p < 0.05. **(H)** Unc5b mRNA levels before and after Tet2 knockdown after Upf1 overexpression were detected by RT-PCR. *n* = 4, *p < 0.05. **(I)** mRNA stability of Unc5b before and after Tet2 knockdown after Upf1 overexpression was detected by RT-PCR. *n* = 6, **p < 0.01.3.2. Quantified data are normalized to the control group, whose value is equal to 1. All data are presented as the mean ± S.E.M. Unpaired two-tailed Student’s t-test was used.

## Discussion

Our previous findings showed that Tet2 protein expression was increased in the mouse hippocampus under chronic mild stress conditions and accumulated in the cytoplasm (Zhang et al., 2021). Some studies have reported that RNA 5hmC modification is highly expressed in the mouse hippocampus and other brain tissues (Miao et al., 2016), but the changes in RNA 5hmC after stress are not clear. In this study, we detected the RNA 5hmC level in the hippocampus of CMS model mice, and the results showed that the level of RNA 5hmC increased after chronic mild stress. Among the Tet family, only Tet2 showed an increase in mRNA and protein levels, while Tet1 and Tet3 decreased at both mRNA and protein levels, suggesting that the increase of cytoplasmic Tet2 may be an important contributor for the increased level of RNA 5hmC. Therefore, in this study, we illustrated that cytoplasmic Tet2 participates in the regulation of mRNA expression through RNA 5hmC modification under stress conditions.

Among the epigenetic modifications, the most widely studied are DNA methylation modification and hydroxymethylation modification (Moore et al., 2013; Zhang et al., 2014). With the advancement of RNA modification identification methods, researchers found that RNA, including tRNA, rRNA, and mRNA, all have RNA methylation modification and hydroxymethylation modification, namely, RNA 5mC and RNA 5hmC (Machnicka et al., 2013; Boccaletto et al., 2018). Studies have reported that RNA 5hmC modifications mainly exist in mRNA (Xu et al., 2016) and are involved in regulating mRNA stability (Lan et al., 2020). Tet enzymes, as the dioxygenase of DNA 5 mC (Tsiouplis et al., 2020), have also been found to act as the hydroxymethylase of RNA 5mC in recent years (Fu et al., 2014; Guallar et al., 2018).

To further confirm the modification of RNA 5hmC by Tet2, we performed Tet2 knockdown in N2a cells using siTet2. The results were consistent with expectations, and the expression of RNA 5hmC was reduced after knockdown of Tet2 and increased by overexpression of Tet2 CD. Taken together, we confirmed that Tet2 is the dominant protein responsible for the increased modification of RNA 5hmC under chronic stress. Studies reported that RNA-modifying enzymes and RNA-binding proteins cooperate in the regulation of transcripts (Boo and Kim, 2020). Here, we found a potential interaction between Tet2 and the RNA-binding protein Upf1 by performing GO analysis on the mass spectrometry data of Tet2 and confirmed their interaction by CO-IP. NMD, which is arguably the best-characterized translation-dependent regulatory pathway in mammals, selectively degrades mRNAs as a means of post-transcriptional gene control (Hug et al., 2016). This control can be used for ensuring the quality of gene expression. Alternatively, such genetic control can facilitate the adaptation of cells to changes in their environment. The key to NMD, irrespective of its purpose, is the ATP-dependent RNA helicase Upf1, without which NMD fails to occur (Brogna et al., 2016; Hug et al., 2016). Subsequently, we found that Tet2 and Upf1 are involved in the regulation of mRNA stability in axonal guidance and neurodevelopmental pathways through complex-mediated RNA 5hmC modification.

In conclusion, we found that increased expression of Tet2 after chronic stress in the cytoplasm led to an increase in RNA 5hmC modification. We, therefore, focused on the role and mechanism of 5hmC modification of RNA under chronic stress. In addition, Tet2 and its new interacting protein Upf1 can participate in the regulation of stress-related mRNA stability in the form of a complex, and the common target genes of Tet2 and Upf1 are mainly involved in axon guidance-related genes, also indicating that neuronal development plays a critical role in chronic stress-related diseases such as depression. However, there are still some gaps in our study, such as where the increase of Tet2 and RNA 5hmC in nerve cells mainly occurs after chronic stress, and other roles of Tet2 on RNA 5hmC modification in chronic stress, which are also the focus of our future research.

## Data Availability

The original contributions presented in the study are included in the article/Supplementary Material; further inquiries can be directed to the corresponding authors.
